The article "Efficacy of Analgesic Propofol/Esketamine and Propofol/Fentanyl for Painless Induced Abortion: A Randomized Clinical Trial" was retracted in 2023. Reasons: signs of a paper mill; compromised peer review; unreliable results or conclusions.

# Efficacy of Analgesic Propofol/Esketamine and Propofol/Fentanyl for Painless Induced Abortion: A Randomized Clinical Trial

**DOI:** 10.1155/2022/5095282

**Published:** 2022-06-09

**Authors:** Naixing Xin, Wei Yan, Shuangfen Jin

**Affiliations:** Department of Anesthesiology, Maternal and Child Health Hospital of Hubei Province, China

## Abstract

**Background:**

Patients have widely accepted abortion as a remedy for contraceptive failure all over the world. Esketamine is a new anesthetic, sedative, and analgesic drug. Fentanyl is an opioid receptor agonist and a commonly used sedative. It is necessary to choose appropriate sedative drugs for painless abortion.

**Methods:**

We selected 238 cases of painless induced abortion from January 2020 to January 2022. We collected surgical parameters, the performance of sedation, and postoperative scales with complications before and after the operation. SPSS 21.0 was used to analyze data.

**Results:**

Surgical indicators between intervention and control groups had no difference; the preoperative indicators including intraoperative bispectral index (BIS), systolic blood pressure (SBP), diastolic blood pressure (DBP), and pulse oxygen saturation (SpO2) had no difference between the two groups. But after surgery, experiment groups had a higher value than the control group in these four indicators. The incidence of postoperative complications including nausea and vomit had no significant difference while the experiment group had a lower *r*-value than the control group in hypotension, bradycardia, decreased oxygen saturation, and respiratory depression. The postoperative VAS score and Ramsay score in the experimental group were lower than those in the control group.

**Conclusion:**

Since esketamine had better sedation performance, reduce the risk of cardiovascular and respiratory depression during sedation, and reduce the pain scale compared with fentanyl, we supported that propofol/esketamine is a good choice for patients receiving a painless induced abortion, and it is a sedation plan worth promoting and further analysis.

## 1. Introduction

Worldwide, abortion is considered one of the main methods of contraceptive failure. According to statistics, there are more than 50 million miscarriages worldwide each year (1). On this basis, countries around the world have adopted various methods to reduce its harm, such as promoting contraceptive knowledge, contraceptive methods, and pregnancy knowledge (2). Even with increased publicity, the number of induced abortions is still increasing, and the incidence of induced abortions shows a clear upward trend (3).

Painless abortion is an abortion with intravenous anesthesia, which adds general intravenous anesthesia to the negative pressure suction abortion procedure to eliminate the patient's physical pain during the procedure and thus gain inner comfort (4). After intravenous administration, the patient falls asleep in about 30 seconds, and the procedure is completed without the pregnant woman's knowledge (5). Several authors have concluded that fentanyl combined with propofol anesthesia has many advantages, such as less pain, no fear, easy administration, and quick postoperative recovery (4, 5). However, previous reports have found that fentanyl combined with propofol anesthesia still has many shortcomings (6, 7). During cervical dilation, most patients exhibit involuntary limb distortions that compromise the surgical outcome, thus greatly increasing the risk of cervical injury. Also, if the dose of propofol is increased, it can lead to significant respiratory depression and circulatory depression (6). In addition, during a painless abortion, the patient's myometrium is in a flaccid state, increasing the incidence of vaginal bleeding, and too many aspirations and scraping are more likely to cause cervical mucosal injury and endometrial basal layer injury (7).

Many scholars have endorsed propofol combined with low-dose fentanyl for intravenous anesthesia (8, 9). Fentanyl, as an opioid receptor agonist, has a rapid onset of action, a short duration of action, and a strong analgesic effect without affecting the patient's normal breathing. When combined with propofol, sedative and analgesic effects are enhanced, and propofol dosage is significantly reduced (10, 11). Esketamine is a novel narcotic sedative and analgesic agent, a derivative of phencyclidine and ketamine, a noncompetitive N-methyl-D-aspartate (NMDA) receptor, and an antagonist. Esmitamine is a dextro structure with a stronger potency in the ketamine family with NMDA receptor affinity and opioid *μ* (12). The receptor affinity is stronger than that of ketamine. The intensity of anesthetic analgesia and hypnosis is twice that of racemic ketamine, while the dose of the same anesthetic effect is only half of the latter (13). The effects of esmitriptamine are more rapid and shorter in duration. It has a high degree of controllability of anesthesia and sedation and analgesia. Esmedetomine has nonrespiratory and mildly excitatory circulatory properties, so it has a more negligible circulatory and respiratory depression than propofol. However, the use of ketamine alone as a sedative analgesic has been limited in the past due to the frequent nausea, vomiting, involuntary physical reactions, and sympathetic stimulation induced by ketamine analogs (14). The combination of esketamine and propofol gives better results. Propofol combined with ketone anesthesia induction has been reported to have good safety and reliability; improve hemodynamics, surgical stress, and inflammatory response; shorten anesthesia time; promote postoperative cognitive recovery; and have less adverse effects (15).

To date, there are limited articles comparing propofol/escitalopram and propofol/fentanyl for painless induction of labor in children, and this article may be the first exploration of this topic.

## 2. Methods and Materials

### 2.1. Design of the Study

In this study, 238 patients from January 2020 to January 2022 were selected. The inclusion criteria were American Society of Anesthesiologists (ASA) female patients with physical status I and II, aged between 20 and 42 years. They were scheduled to have an abortion and required general anesthesia. Exclusion criteria included a history of chronic pain or psychiatric disorders, hepatitis and renal failure, severe metabolic disorders, or cardiovascular disease. Depending on the drug used, patients were divided into an experimental group (esketamine) of 120 and a control group (fentanyl) of 118, both compatible with propofol (Figure 1). The baseline data of the two groups were not statistically significant and were comparable. We compared the clinical effectiveness and safety of the two anesthetic methods.

### 2.2. Anesthesia Methods

All patients were admitted at least one day prior to the procedure, fasted for 24 hours, and water fasted for 8 hours. Oral alprazolam 0.25 mg was administered on the morning of the operation, and intravenous dexamethasone 10 *μ*g/kg, ondansetron 4 mg, and phencyclidine 0.5 mg were administered 20 minutes before the operation. Painless abortion was performed by a senior obstetrician-in-charge, a senior anesthesiologist was responsible for administering anesthesia, and an anesthesiologist was responsible for collecting relevant clinical data.

During anesthesia, the patient was routinely monitored by a multifunctional monitor for ECG, noninvasive blood pressure, pulse oximetry (SpO2), respiratory rate, and bispectral index (BIS) upon entering the operating room. Relevant data were collected and recorded every 5 minutes. We opened intravenous access and infused balanced salt solution at a rate of 4 mL/(kg-h); the patient was placed in a lateral position with the head tilted to the right, and oxygen was administered at a flow rate of 4 L/min through a nasal cannula. For induction medication, fentanyl 1 mg/kg + propofol 1 mg/kg was given to the control group, and propofol 1 mg/K + estradiol 1 mg/kg was given to the observation group with slow intravenous administration (15 min after injection). In the control group, fentanyl 0.5 mg/(kg-h) + propofol 4 mg/(kg-h) was administered intravenously; in the observation group, propofol 4 mg/(kg-h) + estradiol 0.5 mg/(kg-h) was given.

During the operation, we adjusted the dosage of anesthetics according to the BIS value. When the anesthesia was too deep, we reduced the anesthetic agent by 10% each time. At the same time, the anesthetic drug was reduced. After 5 minutes of observation, the attending obstetrician and gynecologist decided to resume or abandon the operation. We treated hypotension and bradycardia by accelerating the infusion rate, intravenous ephedrine 5 mg, or intravenous atropine 5 mg *μ* G/kg. A modified Aldrete score was used as the awake scoring criterion, and scores were recorded every 5 minutes from the end of the procedure with a recovery index of 9 or more. The beginning of induction was defined as the beginning of anesthesia, and the end of maintenance was defined as the end of anesthesia. Complications during and after recovery, such as vomiting, nausea, and shivering, were recorded.

### 2.3. Statistical Analysis

Sample size calculations were based on observational data from our hospital sedation database. Thus, the sample size required for a 15% reduction in need was 120 cases (60 cases per group) with a power of 0.80 and a significance level of 0.05.

Data collection followed the requirements of the prospective intervention study. Data are mean ± SD for continuous variables and number of cases for discontinuous variables. Statistical analysis was performed using SPSS 21.0 (SPSS Inc., Chicago, IL, USA). The student's *t*-test was used for continuous variables, and the Kruskal-Wallis test or Mann–Whitney test was used for nonparametric variables. The Chi-square test and Fisher exact test were used for discontinuous variables. *P* < 0.05 is statistically significant.

## 3. Results

### 3.1. The Baseline Patient Characteristics

The characteristics of the selected subjects are shown in Table 1. 238 samples were recruited from January 2020 to January 2022, and we analyzed the final results. The sample size was 120 cases in the experimental group and 118 cases in the control group. There were no statistically significant differences between the two groups in terms of age, BMI, preoperative heart rate, and mean arterial pressure (Figure 1) (*P* > 0.05).

### 3.2. The Operation Process

As shown in Table 2, we compared the observed indicators between the experimental and control groups. There was no statistically significant difference in anesthesia time between the experimental and control groups (*P* = 0.09). There was no statistically significant difference in operative time between the experimental and control groups (*P* = 0.08). There was no statistically significant difference in recovery time between the experimental and control groups (*P* = 0.45).

### 3.3. The Performance of Sedation and Analgesia

Table 3 shows the hemodynamic and respiratory indices, including BIS, blood pressure, and oxygen saturation, before and after the anaphylactic abortion. Interestingly, there was no statistical difference in mean preoperative heart rate, oxygen saturation, respiratory rate, and arterial pressure between the two groups. However, all four indices were higher in the experimental group than in the control group.

### 3.4. Postoperative Scales and Complication

From Table 4, we can find that the postoperative VAS score and Ramsay score in the experimental group were lower than those in the control group. Hypotension, bradycardia, decreased oxygen saturation, and respiratory depression were lower in the experimental group than in the control group (*P* < 0.05). There was no significant difference in the incidence of nausea and vomiting (*P* > 0.05).

## 4. Discussion

In this study, we found no difference between the two anesthesia protocols during the painless abortion procedure. Before sedation, there was also no difference in the performance of sedation and analgesia between the two groups. However, after sedation, BIS, SBP, DBP, and SpO2 were higher in the experimental group than in the control group. These results suggest that propofol/escitalopram has better sedative and analgesic effects than propofol/fentanyl. In the comparison of complications, hemodynamic and respiratory-related complications were lower in the propofol/escitalopram group than in the propofol/fentanyl group, while digestive-related complications were not statistically different in the two groups. This complication result also suggests that the sympathetic properties of estramustine reduce the risk of cardiovascular and respiratory depression during sedation. In the comparison of pain scales, the experimental group scored lower than the control group, suggesting that propofol/estramustine eliminates postoperative pain.

As the implementation of intravenous anesthesia in painless induction of labor becomes more common, the choice of specific anesthetic drugs has become a focus of clinical attention and research (16). Esketamine is a racemic mixture of S(+)-ketamine and R(-)-ketamine. Esketamine is a right-handed branch of ketamine. It entered the German market in 1997 and was subsequently launched in several European countries (17). It has twice the anesthetic effect of racemic mixtures and is approximately three times more potent than (R)-ketamine. Due to the dose-dependent side effects of ketamine, small doses of esmolol can reduce the incidence of anesthetic side effects (18). Compared with racemic ketamine, esmolol has a lower incidence of psychotropic side effects at equivalent analgesic doses in healthy volunteers, resulting in a rapid recovery with reduced impairment of attention and primary memory capacity (19). The advantages of esketamine are to minimize the side effects of sedation, to make the best use of the concept of synergy, and as an analgesic. It has effective anesthetic and analgesic effects but can still maintain spontaneous breathing and airway reflexes. Hypotension is less common because of increased sympathetic tone (20). Stultz et al. (21) demonstrated that ketamine could improve the quality of sedation and analgesia in patients with difficult sedation in induced abortion (21). They observed a shorter recovery time compared with opioids and benzodiazepine sedation. However, they believe that further randomized trials are necessary. Markus et al. (22) suggested that propofol should be combined with ketamine because of its analgesic effect and no cardiopulmonary inhibition.

Esketamine is not only a well-known sedative but also has a strong analgesic effect. In addition, its sympathetic properties counteract the hemodynamic depressant effects of propofol, thereby reducing the risk of cardiovascular and respiratory depression during sedation (23). However, a potential problem with esketamine may be its mental analog effects, such as visual impairment, nausea, or vertigo, affecting patient satisfaction (24).

When esketamine is used as a single sedative, it is limited by its psychotropic and vomiting-inducing effects. Compared to the target-controlled infusion (TCI) with propofol and ketamine sedation, the patient's propofol dose can be reduced by 15% under the same sedation conditions (25). Some experts believe that esketamine can replace opioids as a contraction additive to propofol sedation because propofol can be used in smaller amounts with limited cardiopulmonary side effects to achieve adequate levels of sedation and analgesia (26). Therefore, the total amount of propofol is an option for the effectiveness of sedation adjuvants.

In addition, Nan et al. found that propofol combined with low-dose ketamine for monitored anesthesia during surgery reduced propofol-induced hyperventilation, induced stable positive spirits, and allowed earlier recovery of consciousness compared to propofol alone (27). However, the most common suspicion is the cognitive alteration effect of estaminet, which can produce a psychotomimetic effect similar to schizophrenia (28). On the other hand, Karkare et al. (29) have shown that clinically relevant doses of propofol inhibit these effects by activating GABA receptors. Therefore, the pharmacokinetics and pharmacodynamics of esketamine in combination with propofol need further investigation (30).

In summary, we conducted a randomized controlled trial to compare the clinical efficacy and safety of propofol/esketamine and propofol/fentanyl groups. According to the results, the two sedation regimens did not differ significantly in terms of the abortion procedure and procedural safety. However, propofol/esketamine showed better results than propofol/fentanyl in terms of hemodynamics and respiratory function and related complications. Therefore, we believe that propofol/estradiol is a good choice for patients undergoing painless induction of labor and is a sedation regimen worthy of promotion and further analysis.

## Figures and Tables

**Figure 1:** Patient randomization in the trial.

**Table 1:** Demographic and clinical characteristics of each study group.

Variable	Experiment (*n* = 120)	Control (*n* = 118)	*t* value	*P* value
Age (years)	27.25 ± 2.32	27.19 ± 1.21	0.25	0.80
BMI	20.72 ± 3.63	20.25 ± 3.36	1.04	0.30
Heart rate	81.85 ± 6.85	80.52 ± 7.58	1.42	0.16
Mean arterial pressure	85.52 ± 10.85	87.28 ± 11.81	-1.20	0.23

**Table 2:** Surgical parameters of each study group.

Variable	Experiment (*n* = 120)	Control (*n* = 118)	*t* value	*P* value
Duration of anesthesia (min)	6.82 ± 1.72	6.51 ± 1.01	1.69	0.09
Duration of surgery (min)	186.85 ± 22.85	181.52 ± 23.58	1.77	0.08
Time to wake up (min)	6.25 ± 2.25	6.02 ± 2.48	0.75	0.45

**Table 3:** Performance of sedation and analgesia in each study group before and after surgery.

Variable	Experiment (*n* = 120)	Control (*n* = 118)	*t* value	*P* value
Preoperative				
BIS	96.48 ± 2.65	96.37 ± 2.25	0.35	0.73
SBP	110.82 ± 10.75	110.63 ± 10.74	0.14	0.89
DBP	73.67 ± 6.88	74.15 ± 6.16	-0.57	0.56
SpO2 (%)	99.85 ± 1.98	99.52 ± 1.35	1.50	0.14
Postoperative after 15 min at recovery				
BIS	84.01 ± 1.95	74.25 ± 1.82	39.9	<0.01
SBP	111.23 ± 11.92	99.35 ± 6.42	9.55	<0.01
DBP	73.13 ± 6.18	64.72 ± 2.52	13.71	<0.01
SpO2 (%)	98.38 ± 0.85	87.64 ± 1.25	77.63	<0.01

^∗^BIS: intraoperative bispectral index; SBP: systolic blood pressure; DBP: diastolic blood pressure; SpO2: pulse oxygen saturation.

**Table 4:** Recovery and complications of each study group.

Variable	Experiment (*n* = 120)	Control (*n* = 118)	*χ* ^2^/*t* value	*P* value
VAS score	2.85 ± 0.62	3.91 ± 0.81	-11.35	<0.01
Ramsay score	2.25 ± 0.51	2.68 ± 0.63	-5.73	<0.01
Hypotension	2	12	6.31	0.01
Bradycardia	3	12	4.69	0.03
Movement	5	17	6.27	0.01
Respiratory depression	1	9	5.24	0.02
Nausea and vomit	5	6	0.01	0.97

## Data Availability

No data were used to support this study.
